# Optimization and Simulation of Manuscript Management System Based on Fuzzy Genetic Neural Network

This article has been retracted.

**DOI:** 10.1155/2021/3155765

**Published:** 2021-08-17

**Authors:** Yongtai Sun

**Affiliations:** Editorial Department of Journal, Jimei University, Xiamen 361021, China

## Abstract

Manuscript management plays an important role in the whole periodical industry. Journals and magazine society receive different types of contribution documents from all over the world. Many submission files are mostly transmitted by e-mail, but there are some hidden disadvantages in e-mail. In view of this situation, this paper studies the establishment and optimization simulation of manuscript management system based on fuzzy genetic neural network (FGNN). On the basis of genetic neural network, combined with the advantages of FNN neural network algorithm, a FGNN structure is established to optimize the system, which is helpful to the learning and expression ability of the whole system. The results show that the FGNN can extract and express the structured data, and the submission management system runs faster. Then, UML modeling and PHP framework are used to realize the design and establishment of the system, and the simulation model of contribution system is constructed. The innovation of this study is to combine genetic neural network with FNN neural network, which can query, manage, and classify manuscripts quickly. It also improves the complex submission system and optimizes the submission process. The whole journal editing work has been effectively improved.

## 1. Introduction

As one of the important tools to publicize cultural and scientific information, journal manuscripts have always been in a very popular position in the process of knowledge dissemination and cultural innovation [1]. In the context of the annual sustained growth of manuscripts, the types of manuscripts are becoming more and more colorful [2]. It is very important to establish an effective and convenient system of contribution rules for the collection and management of contributions. The traditional way of contribution can only meet the needs of a small number of people [3, 4]. At present, with the progress of science and technology and the development of computer science, people's demand for contributions has gradually become higher and higher. The traditional way of contribution has a certain degree of backwardness, which is not helpful to the editing and management of the whole manuscript [5, 6]. This way also leads to the decrease of the work efficiency of journal editors, magazines, and other organizations, and the information can not be obtained and used at the first time, seriously hindering the dissemination and development of information resources [7]. And this kind of information lag and poor compatibility situation can not meet the rapid development of information society. How to change the time of manuscript acquisition and review and improve work efficiency is a problem that every journal editing department needs to face [8]. How to improve the management of contributions, effectively review contributions, and edit contributions and other work is the daily need of journal editorial departments to consider [3]. With the rapid development of the Internet, the speed of information dissemination is also faster and faster. If we cannot solve the problem of contribution, it will reduce the work speed of the whole editorial department [9, 10]. In the face of this need to quickly process a large number of manuscripts and classify manuscripts in real time, it has become a problem that journal workers need to quickly solve [11]. So it is very important to realize the management optimization and simulation model construction of contribution system. It can release most journal workers from useless repetitive work and have more time to deal with other work [12].

In the framework of automatic intelligent contribution system, the advantages and efficiency of the contribution system should be reflected [13]. Its purpose is to liberate the repetitive work of editors and improve the whole journal and editing and publishing process. Neural network is mainly based on the continuous optimization of network structure system to realize the training model. For the research on the principle and construction model of the whole neural network system, the neural unit in the neural network is analyzed first [14]. In the presence of neural units, the final network structure is formed through model reorganization and training. In the neural network model, we mainly start from two aspects [15]. They are artificial neural network structure and unit neural model. The unit neural network in the structure of artificial neural network is necessary for the topology construction of the whole network. When the network structure definition is reorganized, the joint weight value is carried out according to the structure of the network topology to change the various functions of the artificial neural network structure [16]. At present, neural network algorithms and network structure models have been generated from many kinds of optimization. These new neural network algorithms have achieved excellent results in various fields [17]. Sun et al. established the minimum levitation unit of maglev vehicle system. An amplitude saturation controller (ASC) is proposed, which can ensure that only saturated unidirectional attraction is generated. The stability and convergence of the closed-loop signal are proved based on Lyapunov method [18]. In recent years, neural network algorithm can monitor the action trajectory of maglev train in delayed rail transit and solve the problem of intelligent transportation. In the medical field, medical images can also be processed according to neural network algorithm. Genetic algorithm can improve its own organizational structure and complex data set problems according to mechanism problems. It is an automatic complex neural network algorithm model, which can accurately deal with the construction problem of complex data information [19]. These new neural network algorithm structures have different characteristics and functions in the whole network topology, learning and training methods, activation function properties, and so on [20]. Fuzzy neural network is a kind of network structure which is different from other neural network algorithms. It can express the time change rule and structure of continuous range. The main structure is also different from ordinary neural network algorithm, including input data layer, fuzzy calculation layer, rule establishment layer, normalization processing layer, propagation layer, and output data layer [21]. Through the structure of fuzzy neural network, it can be seen that if the algorithm is used in the manuscript management system, it can complete the overall planning and training control of the system efficiently. Sun et al. [22] proposed a semisupervised controller based on deep belief network (DBN) algorithm in the presence of unknown external interference. This method can effectively deal with the unmeasurable air gap velocity and generalized external interference and ensure the vertical safety of the output air gap in a certain range.

Both neural network structure and fuzzy algorithm can be used for data analysis and model prediction [23]. Mehta et al. [24] designed an adaptive robust controller using Riccati method and sliding mode technology, taking into account the effects of time delay and disturbance. The asymptotic stability of the closed-loop system is proved by Lyapunov method. The simulation results show the control performance of the controller. It can realize the construction of the system which can deal with the problems and distributed processing, data storage, and other functions. Fuzzy neural network unifies the advantages of itself and genetic neural network algorithm and improves the learning and training function and representation and storage function of the whole system [25]. In the construction of management system, the problems of coupling and information combining are not smooth, which can be well solved by using FGNN algorithm. So this algorithm has been widely concerned in today's neural network algorithms. With the selection of algorithm, in order to establish the simulation model of the whole contribution system, we also need to select the modeling method [26]. Xia et al. proposed a fast and accurate analysis method of maglev vehicle bridge system to analyze the influence of bridge and controller on the dynamics of maglev system [27]. In the software system structure design, whether the system structure modeling can reflect the overall function and accuracy determines whether the whole system has development significance. For the modeling of contribution system, we use unified modeling language (UML) to build object-oriented language. The realization of visual modeling function can provide solutions from different perspectives for the whole system.

This paper first analyzes and discusses the traditional way of contribution and concludes that there are some defects in the traditional way of contribution. According to this situation, a technical model based on FGNN is constructed for research, and the network structure of contribution system is established by combining with FNN basic algorithm. Then we use PHP language and UML modeling technology to build the manuscript management system and realize the simulation model. The model of manuscript management system based on FGNN and simulation is analyzed.

## 2. Research on the Establishment Technology of Manuscript Management System Based on FGNN and Modeling

### 2.1. Research on Basic Neural Network Technology Based on FGNN and FNN

The traditional way of e-mail submission will be used in the use of journal departments and conferences. But the defect of e-mail contribution is also very obvious and more and more prominent [28, 29]. Journal workers need to register, mark, typeset, and check the manuscripts. When the information is incomplete, they need to process the whole manuscript immediately. If it is not handled in time, it will lead to serious problems such as delayed publication of the whole journal. In order to better face the problem of a large number of manuscript sources and the work efficiency of editors, we build a manuscript management system based on FGNN algorithm. Before building the system model, we first analyze the structure of FGNN. The model is shown in Figure 1.

The whole neural network structure is mainly divided into five layers, which are fuzzy input data layer, fuzzy process layer, condition layer, decision layer, and fuzzy elimination output data layer. If the variable parameters in the whole FNN system are output data object and input data object, respectively, then two fuzzy network subsets are generated in the network structure. In the input data layer, nodes are represented as input data object parameters to sort the network hierarchically. After the input data is integrated, it enters the fuzzy layer through membership function. The function formula is as follows:

(1) $$\begin{array}{c} I_{j}^{2}=w_{ij}^{2}o_{i}^{1};\\ o_{j}^{2}=f\left(i_{j}^{2}\right). \end{array}$$

After entering the fuzzy level, the defined requirements in the rules are combined and matched to form the multiplication operation between the fuzzy parameters of the input data. The actual formula is as follows:

(2) $$\begin{array}{c} I_{t}^{3}=\prod_{j}w_{jl}^{3}o_{i}^{2};\\ o_{t}^{3}=I_{t}^{3}. \end{array}$$

The range of fuzzy degree of corresponding output data node value is obtained

(3) $$\begin{array}{c} I_{K}^{4}=\sum_{t}w_{lk}^{4}o_{t}^{3};\\ o_{k}^{4}=\min\left(1,I_{k}^{4}\right). \end{array}$$

In the last layer, the fuzzy value of the output data is removed, and the parameters of the output fuzzy data variable are restored and displayed in the form of multiplier

(4) $$\begin{array}{c} I^{5}=\sum_{k}w_{kl}^{5}o_{k}^{4}=\sum_{k}\left(m_{k}\sigma_{k}\right)o_{k}^{4},\\ y=o^{5}=\frac{I^{5}}{\sum_{k}\sigma_{k}o_{k}^{4}}. \end{array}$$

In the formula, the number of neural units at each level is expressed as input data by variables. The number of output data neural units of each level is also defined. Finally, the center of membership function and the range width are calculated. In the construction of the prediction model of the system, the genetic algorithm is used to optimize the fuzzy neural network system. The internal structure of this model includes the number of nodes in the whole hidden layer and the value of membership function variables, that is, the number of central layers of the neural network structure, the central value of the function, and the range width. The operation flow of FGNN is shown in Figure 2.

We normalize the input data samples of the whole network model in order to reduce the impact of data information on the construction and prediction of the whole system. The real-time data is normalized and transformed into functions. The formula is as follows:

(5) $$\begin{array}{c} y=\frac{\left(y_{\max}-y_{\min}\right)*\left(x_{\max}-x_{\min}\right)}{x_{\max}-x_{\min}}+y_{\min}. \end{array}$$

In the formula, variables are defined for the maximum and minimum values, which, respectively, represent the size range of the input data. After that, unified planning was carried out. The initial network structure parameters are set in advance, and the number of hidden layer nodes is counted. After the membership function is calculated, the training evolution is carried out according to the size of the population. Get all the evolution update times. Test the crossover probability and mutation probability of the model. We use big data statistics for data acquisition and get all the data models and feature points in the total sample. The sample includes marking and analyzing the source, type, time, and other aspects of the manuscript and calculating the parameters as input data information variables. The overall data obtained form a data set and are stored in the database. After establishing the model, we need to verify the performance of the whole system model and use the arithmetic root mean square error, absolute error, and percentage error to analyze and summarize the system model.

With the development of science and technology, the system for the need to control the parameters and objects has gradually increased to one to many mode. Because of the complexity of the system, the parameters of variables are interrelated. Therefore, we need to build a multivariable object system model for a large number of inputs and outputs of submission data. The characteristic of multivariable object system model lies in the joint reaction between input data and output data. It is difficult to get accurate model, so we can use SISO system to replace the same level system. In order to improve the operation speed and representation ability of the whole system and to solve the problem of data repeatability, we first use genetic algorithm to optimize the membership function, center value, and weight value of FNN model algorithm. FNN combines the whole system with neural network to form the training ability of connection structure. The changes of membership function, center value, and weight value before and after optimization are shown in Figure 3.

It can be seen from Figure 3 that the optimized values can solve the problem of data repeatability and improve the system performance. FNN structure is divided into input data layer, which can transfer numerical variables to the next layer. The number of nodes and the input variable parameters are connected, respectively. In the second layer, the membership function of the parameters is calculated. The formula is as follows:

(6) $$\begin{array}{c} \mu_{i}^{j}=\mu_{Ai}^{j}\left(x_{i}\right). \end{array}$$

The formula used in the segmentation of membership function is as follows:

(7) $$\begin{array}{c} \mu_{Ai}^{k}\left(x_{i}\right)=\exp\left[-{\left(\frac{x_{i}-a_{i}^{k}}{a_{i}^{k}}\right)}^{2}\right]. \end{array}$$

After the membership function is calculated, the center value and data range width are expressed:

(8) $$\begin{array}{c} N_{2}=\sum_{i=1}^{n}m_{i}. \end{array}$$

The fitness is adjusted according to the calculated system rules:

(9) $$\begin{array}{c} a_{j}=\min\left\{\mu_{1}^{i_{1}},\mu_{2}^{i_{2}},\ldots ,\mu_{n}^{i_{n}}\right\}. \end{array}$$

Finally, the normalization calculation is carried out, which is clear with the output data layer. The number of nodes should be consistent with the upper layer. The formula is as follows:

(10) $$\begin{array}{c} \bar{a}=\frac{aj}{\sum_{j=1}^{m}aj},\;j=1,2,\ldots ,m,\\ y_{i}=\sum_{j=1}^{m}w_{ij}\bar{a_{j}},\;i=1,2,\ldots ,r. \end{array}$$

In order to solve the problem of data duplication in a variety of input and output data systems, we carry out the operation of deduplication method. The purpose is to realize the function of efficient, clear, and simple contribution system. This operation structure will not affect the characteristics of the control process. It can simplify the whole system.  Figure 4 shows the operation rate of data system with and without deduplication.

It can be seen from Figure 4 that the system operation rate has been significantly improved after the problem of duplicate data is eliminated. The FNN algorithm model used has multiple neural units, and the output data parameters are transformed into fuzzy function. The formula for solving the problem of data duplication is as follows:

(11) $$\begin{array}{c} l_{12}=\sum_{j=1}^{m\left(1,2\right)}w_{ij}^{\left(1,2\right)}{\overset{-\left(1,2\right)}{a}}_{j},\\ l_{13}=\sum_{j=1}^{m\left(1,3\right)}w_{ij}^{\left(1,3\right)}{\overset{-\left(1,3\right)}{a}}_{j},\\ l_{21}=\sum_{j=1}^{m\left(2,1\right)}w_{ij}^{\left(2,1\right)}{\overset{-\left(2,1\right)}{a}}_{j},\\ l_{23}=\sum_{j=1}^{m\left(2,3\right)}w_{ij}^{\left(2,3\right)}{\overset{-\left(2,3\right)}{a}}_{j},\\ l_{31}=\sum_{j=1}^{m\left(3,1\right)}w_{ij}^{\left(3,1\right)}{\overset{-\left(3,1\right)}{a}}_{j}. \end{array}$$

According to the feedback mechanism, the above formula forms a matrix formula to remove data repetition. When the FGNN algorithm is selected, the initialization value is given according to the parameters and variables. Then the transmission rate of each system channel is detected. If the function of eliminating duplication is realized, the output data value will appear in the expected effect. So the formula of FNN to solve the repetition problem is shown above. In the learning and training process of the whole system, it is necessary to improve the running speed of FNN to optimize the system. The process of obtaining membership function and center value range of fuzzy algorithm improved by genetic neural network is as follows: firstly, the branch rules of network structure system are selected to determine the range and width of membership function. There will be random parameter variable values in the range, and different parameter populations will be formed according to the variables. Finally, the parameter selection and crossover mutation operation are carried out for the whole neural network system. After the analysis of the error results, the whole learning and training is finished, and the output data value is obtained.

### 2.2. Design and Implementation of Contribution System Based on UML and PHP Framework

In the design of contribution system, we should first analyze the contribution methods, mainly using the registration method to obtain user information. It is also convenient for the management and classification of the whole manuscript owner information. When browsing the contribution, it can divide the contribution according to the data information, which is convenient for query and storage. In order to reduce the workload of the whole contribution system, we also need to consider reducing the number of duplicate uploads, preprocessing and eliminating the duplicate overlapped manuscripts. In the traditional management mode, we can only query the source of contributions without personal information by person-to-person telephone or e-mail. The corresponding writers can only make inquiries in the process of reviewing manuscripts by traditional means such as calling. When unable to deal with the remaining problems in time, the manuscript makes the whole workload more and more. We need to design a real-time contribution system that can automatically manage the classification and query of contributions. However, the automatic classification does not mean that the information can be modified at will. In the construction of the whole system, we need to design the background database, because the establishment of the database can facilitate the query and security of the whole system. An excellent database can help the system improve efficiency and optimize the working mode. It mainly includes user form, author information, time, source address, etc. The preliminary system architecture is shown in Figure 5.

Each framework of the system has different functions, and the modules are interrelated. The contributor module can support online registration editing for the whole process of contribution system and enter the page to submit and edit the content on the page. The manager module is used by the editor to view and manually classify the transmitted manuscripts. At last, we design the evaluation link of the system to evaluate and modify the uploaded manuscript. The key technology is PHP open source framework compiler language, which can render the front-end interface and connect the database of the whole system as a function link. The advantage of PHP framework is that it supports database connection of many modes and rich interface content, which can form fast and effective system functions. Then PHP framework can reduce the cost of background technology development and front interface technology. The schematic diagram of system function module is shown in Figure 6.

With the preliminary framework construction of the system, we need to carry out visual simulation modeling to realize the system architecture. This paper introduces the whole framework process of the system and explains the functions of the key modules. The requirements and framework model of the database are also designed. Then we need to establish a multilevel web framework to ensure the smooth operation of the system. We need to preset the architecture of the framework.

According to the framework and database structure, the server can make the system have a good running environment. We will need to publish the contribution information saved, according to the program that can extract the relevant information of contributors. This new function module can support the server to obtain the content of real-time dynamic data. The requirement information and UML configuration of the whole system model are shown in Figure 7.

After setting web framework and UML parameters, we predict the response speed of the system before and after construction. The prediction is based on input and output indicators, as shown in Figure 8.

## 3. Analysis of Optimization Simulation Results of Manuscript Management System Based on FGNN and UML Modeling

### 3.1. Analysis of Experimental Results Based on FGNN and FNN Neural Network

In this paper, fuzzy neural network combined with genetic algorithm neural network technology is used to build the system framework and simulation model of manuscript management function. This paper mainly analyzes the main influencing factors in the process of submission and the obstacles of calculation running time to the whole system. These factors will make the calculation more difficult and affect the evaluation and prediction accuracy of the system. The data information we use is obtained through random samples, and the simulation operation is realized through the system test function. The source, type, address, time, and other parameters of contributors are input into the system as test data. Firstly, the data effect of the training results of the FGNN algorithm is compared with that of the traditional neural network algorithm, as shown in Figure 9.

Then the training and learning sample data are compared with the expected prediction model data. Analyze the functionality of the whole system. Input the test data into the prediction model to get the output data rate of the prediction system, and compare with the model before FGNN optimization. The comparison data is shown in Figure 10.

From the comparison results, we can see that the actual speed of the calculation process is lower than the estimated effect, but it is very close to the expected data value. This also proves that the FGNN plays a role of optimizing the system in the construction of manuscript management system and can effectively improve the whole operation environment and output results of the system.

Then we analyze the results of FNN algorithm in data processing. FNN algorithm can judge the actual effect according to the reference model when it is used to process the duplicate manuscript data information. By comparing the amount of input manuscript data and the speed of querying manuscript, this paper analyzes whether this algorithm has good influence factors. According to the periodic analysis of the collected data, we can get the conclusion that when the duplicate data is separated, the input manuscript data is taken as the unit quantity, and whether the duplicate manuscript is separated or deleted is analyzed by judging the transmission rate. The experimental results show that FNN algorithm is suitable for multidata input system. It can automatically complete the target requirements without manual intervention of the whole operation and improve the system construction environment and parameter variable input. It improves the accuracy and efficiency of manuscript management.

### 3.2. Simulation Results Analysis of Manuscript Management System Optimization Based on UML Modeling

In the whole environment of system construction, we need to test and try the server. In case of achieving different time and place, different users can carry out manuscript management operation. The main technical analysis includes the technical analysis of the uploaded manuscript, the type separation, and file size compression of the corresponding manuscript in the background. It can improve the manuscript flow speed in manuscript management and facilitate workers to quickly obtain the target manuscript. After analyzing the online preview and dynamic transmission technology in the submission system, the system function created by the compiled language needs to support the online browsing function of the whole submission system. It is convenient for the editorial department to review the manuscript without secondary retrieval. This function reduces the secondary operation of the system and improves the work efficiency of the whole environment. Dynamic dissemination of information is also an important part of manuscript management, mainly to help managers contact contributors. In the process of connecting the web framework and database, we can use character encoding to solve the problem of garbled code.

The system uses the view model to separate and build the input data, processing data, output data, and other processes. The whole system is modeled by UML, and the simulation plane is shown in Figure 11.

Therefore, the architecture of the whole system is not single but is composed of multilayer web framework model. The requirement module is divided into user module, manager module, and audit operation module. It can achieve online delivery and management functions. We use UML to build a simulation model to represent the case of online contribution. In the main category variables of manuscript management system, user, article, operation, editing, access, and other functions are related to each other and marked in the contribution. This simulation model can quickly call manuscripts for optimal management.

## 4. Conclusion

In this paper, through the analysis of the traditional way of contribution, it is concluded that the traditional way of contribution will make the manuscript management more difficult. In order to improve this situation and improve the efficiency of the whole manuscript management, we use the method of manuscript management based on FGNN. Then, the analysis of the research results shows that the FGNN can improve the speed of data acquisition and manuscript processing and classification through the training model. Finally, compiled language is used to build the whole system framework, and UML is used to build the system simulation model. Simulation of the operating environment and process of the system, using UML construction sequence for detailed design, shows the operation process of the entire submission system. Compared with the traditional system without fuzzy genetic neural network, the algorithm used in this paper can reduce the unnecessary steps in the submission process, improving the running speed of the whole system.

## Figures and Tables

**Figure 1:** Structure diagram of FGNN.

**Figure 2:** Operation flow chart of FGNN.

**Figure 3:** The change chart of membership function, center value, and weight of the model before and after optimization.

**Figure 4:** Operation rate of data system with and without duplication.

**Figure 5:** The preliminary system structure frame diagram.

**Figure 6:** Schematic diagram of system function module.

**Figure 7:** Requirement information and UML configuration diagram of system model.

**Figure 8:** Response speed prediction chart before and after system construction.

**Figure 9:** Algorithm training effect comparison chart.

**Figure 10:** Actual output rate vs. expected.

**Figure 11:** UML modeling and simulation system interface.

## Data Availability

The data used to support the findings of this study are available from the corresponding author upon request.
